The article "Identification and Validation of an Inflammatory Response-Related Polygenic Risk Score as a Prognostic Marker in Hepatocellular Carcinoma" was retracted in 2023. Reasons: suspected computer-generated content; unreliable results or conclusions; concerns about the data; concerns about the results or conclusions.

# Identification and Validation of an Inflammatory Response-Related Polygenic Risk Score as a Prognostic Marker in Hepatocellular Carcinoma

**DOI:** 10.1155/2022/1739995

**Published:** 2022-09-28

**Authors:** Huang Xiaochun, Pang Feixiong, Ou Shengsong, Wei Xiaojiao, Xu Yuju, Lai Yanhua

**Affiliations:** ^1^Guangxi Academy of Medical Sciences, Nanning, Guangxi, China; ^2^Department of Transplantation, People's Hospital of Guangxi Zhuang Autonomous Region, Nanning, Guangxi, China

## Abstract

**Aims:**

We hypothesized that the expression patterns of inflammatory response-related genes may be a potential tool for hepatocellular carcinoma (HCC) risk scoring.

**Background:**

Inflammatory response plays a pivotal role in the pathogenesis of HCC.

**Objective:**

To establish and validate a hallmark inflammatory response gene-based polygenic risk score as a prognostic tool in HCC.

**Methods:**

We screened differentially expressed inflammatory response genes and established an inflammatory response-related polygenic risk score (IRPRS) in an HCC-related dataset. Patients with HCC were categorized into high- and low-risk groups according to the median IRPRS, and the overall survival between the two groups was compared. The IRPRS was validated in an independent external dataset. Tumor-infiltrating lymphocytes (TILs) in high- and low-risk groups were compared, and gene set enrichment analysis was performed to characterize high-risk HCC identified using this IRPRS.

**Results:**

Four differentially expressed hallmark inflammatory response genes (*CD14*, *AQP9*, *SERPINE1*, and *ITGA5*) were identified to construct the IRPRS. Patients in the high-risk group had significantly shorter overall survival than those in the low-risk group in both the training set and the test set. Furthermore, the IRPRS remained an independent prognostic factor compared to the routine clinicopathological characteristics. Many cancer-related hallmark gene sets and TILs were significantly enriched in the high-risk group.

**Conclusions:**

We established and validated a four-hallmark inflammatory response gene-based polygenic risk score, which could successfully divide patients with HCC into high-risk and low-risk groups. These two risk groups of HCC possess significantly distinct prognostic and biological characteristics.

## 1. Introduction

The growing incidence of liver cancer and its poor prognosis make it a global health challenge [1]. Hepatocellular carcinoma (HCC) is the most common type of liver cancer accounting for approximately 90% of all cases of liver cancer [2]. The estimated median overall survival (OS) of patients with untreated HCC (all stages) is approximately nine months [3]. In the recent years, we have witnessed considerable advances in the understanding of the molecular pathogenesis and heterogeneity of HCC; however, owing to persisting knowledge gaps, there has been limited application of this knowledge in clinical practice. Development of methods to identify the subset of patients who are at high risk and who may benefit from more active treatment is a key imperative.

In various cancers, there is evidence for the roles that local immune response and systemic inflammation have in the development of tumors and prognosis of patients with cancer. This knowledge provides an opportunity to identify the biomarkers of inflammatory responses to predict patient outcomes [4]. The majority of HCCs occur in the context of chronic inflammation and in the backdrop of a fibrotic liver, with numerous cases associated with hepatitis virus infection, toxins, and fatty liver disease [1, 5, 6]. There is clear evidence showing that inflammation can promote the development of HCC [7, 8]. Moreover, the liver is also an immunologic organ in itself [9, 10], which may enhance the inflammatory response to cancer arising within it. Therefore, we hypothesized that the expression patterns of inflammatory response-related genes may be a potential tool for HCC risk scoring. To assess our hypothesis, we analyzed an HCC-related dataset from the Gene Expression Omnibus (GEO) database and established an inflammatory response-related polygenic risk score (IRPRS), which was validated in another independent dataset.

## 2. Materials and Methods

### 2.1. Data Processing

The 200 inflammatory response hallmark genes were obtained from the Molecular Signatures Database [11, 12]. The processed gene expression profiles in GSE14520 [13] based on Affymetrix HT Human Genome U133A Array (Affymetrix; Thermo Fisher Scientific Inc., Waltham, MA, USA) and prognosis data were downloaded from GEO (https://www.ncbi.nlm.nih.gov/geo) for analysis; the dataset contains data pertaining to 225 HCC and adjacent tissues of HCC patients. The GSE14520 was used to screen the differentially expressed inflammatory response hallmark genes and establish a polygenic risk score. Another HCC dataset (known as TCGA-LIHC dataset) containing RNA sequencing (RNA-seq) data (displayed as raw counts) and clinical information belonging to The Cancer Genome Atlas (TCGA) Program was downloaded from the Genomic Data Commons Data Portal (https://portal.gdc.cancer.gov/) and used to validate the polygenic risk score. The RNA-seq data were normalized by quantile method using *voom* function from limma package [14] in R. When one gene matched multiple probes, the average value of the probes was estimated as the expression of the corresponding gene. Given that GSE14520 has more adjacent tissues, which would be beneficial for identifying differentially expressed genes, it was used as the training set.

### 2.2. Screening Differentially Expressed Genes and Bidirectional Hierarchical Clustering

The expression profiles of the hallmark inflammatory response genes were extracted from GSE14520 and subjected to screen differentially expressed genes in HCC compared to adjacent tissue using limma package. Genes with a *P* value (adjusted by false discovery rate) < 0.05 and ∣fold change | >1.5 were considered as significant. Bidirectional hierarchical clustering to identify the differentially expressed genes based on Euclidean distance was performed and the results displayed as a heat map.

### 2.3. Least Absolute Shrinkage and Selection Operator (LASSO) Cox Analysis

The LASSO Cox regression can be used for the optimal selection of features in high-dimensional data with a strong predictive value and low correlation between each other to prevent overfitting [15, 16]. The expression profiles of differentially expressed hallmark inflammatory response genes were subjected to LASSO Cox analysis with 10-fold cross-validation using the glmnet package [17]. The IRPRS was created using the formula

(1) $$\begin{array}{c} \text{IRPRS}=\text{Expressio}{\text{n}}_{\text{Gene}1}*\text{Coefficien}{\text{t}}_{1}+\text{Expressio}{\text{n}}_{\text{Gene}2}*\text{Coefficien}{\text{t}}_{2}+\cdots +\text{Expressio}{\text{n}}_{\text{Gene}n}*\text{Coefficien}{\text{t}}_{n}. \end{array}$$

“Gene” was the optimal feature with a nonzero coefficient, and “Coefficient” represents its corresponding coefficient. The PRS was calculated for each individual patient, and patients were categorized into high- and low-risk groups based on the median score. Overall survival (OS) was compared between the two groups.

### 2.4. Validation of the Differential Expression and the IRPRS

The validation comprised two parts. First, the differential expression of the optimal feature with a nonzero coefficient was validated in the TCGA-LIHC dataset. In the second part, similar to that in the GSE14520, IRPRS was calculated for all individuals in the TCGA-LIHC dataset using the above formula, followed by their categorization into high- and low-risk groups according to the median score. Furthermore, the TCGA-LIHC dataset contains other routine clinicopathological characteristics; multivariable Cox regression analysis was performed to assess the association of IRPRS with these characteristics.

### 2.5. Gene Set Enrichment Analysis (GSEA)

GSEA [11, 18] was performed to determine the potential biological characteristics of the high-risk HCC identified by the IRPRS. The normalized gene expression profiles of HCC samples from the TCGA-LIHC dataset and the hallmark gene sets were applied to perform GSEA using the GSEA java software. FDR < 0.25 and nominal *P* value < 0.05 were considered significant.

### 2.6. Correlation between the IRPRS and Glypican 3 (GPC3)/HSP70/Glutamate-Ammonia Ligase (GLUL)

GPC3, GLUL (also known as glutamine synthase (GS)), and HSP70 have been identified as robust diagnostic biomarkers [19, 20] and even therapeutic targets for HCC [21, 22]. Thus, we explored the correlation of the IRPRS with these biomarkers. The genes included in the HSP70 family were obtained from a previous study [23]. The mean expression level of these HSP70 genes was used for correlation analysis.

### 2.7. Comparison of Tumor-Infiltrating Lymphocytes (TILs) in the High- and Low-Risk Groups

Tumor-infiltrating lymphocytes (TILs) play a pivotal role in the pathogenesis of HCC [24]. In the present study, the xCell [25] web tool (https://xcell.ucsf.edu/) with Charoentong signature [26] was used to estimate the enumeration of TILs from HCC tissue expression profiles of TCGA-LIHC dataset. Subsequently, we compared the enumeration of TILs in high- and low-risk groups. *P* value (adjusted by false discovery rate) < 0.05 was considered as significant.

### 2.8. Statistical Analysis

All analyses were performed using the R software (version 4.0.2) (https://www.r-project.org/). The unpaired *t*-test provided by limma package was used to compare the gene expression levels and the enumeration of TILs. Kaplan-Meier survival analysis with log-rank method was used to compare OS between groups. The Wilcoxon test was used to compare the IRPRS between groups. Spearman correlation analysis was performed to explore the correlation between two variables. All tests were two-sided and *P* ≤ 0.05 were considered indicative of statistical significance, unless otherwise stated.

## 3. Results

### 3.1. Multiple Hallmark Inflammatory Response Genes Showed Distinct Expression Patterns in HCC Compared to Nontumor Liver Tissue

Thirty-two hallmark inflammatory response genes were found to be differentially expressed in HCC compared to nontumor liver tissue, including 22 downregulated and 10 upregulated genes (Figure 1(a)). The expression patterns of the differentially expressed hallmark inflammatory response genes could distinguish HCC and nontumor tissue (Figure 1(b)).

### 3.2. Four Hallmark Inflammatory Response Genes Constituted the IRPRS

After LASSO Cox analysis, four hallmark inflammatory response genes (*CD14*, *AQP9*, *SERPINE1*, and *ITGA5*) were identified as nonzero coefficient features (Figure 2(a)). IRPRS = expression_CD14_∗(−0.16244) + expression_AQP9_∗(−0.00822) + expression_SERPINE1_∗0.21430 + expression_ITGA5_∗0.09635. Patients in the high-risk group had significantly shorter OS than those in the low-risk group (hazard ratio = 1.026, 95%confidence interval = 1.741–4.470, *P* < 0.001, Figure 2(b)).

### 3.3. Validation of IRPRS in the TCGA-LIHC Dataset

In the TCGA-LIHC dataset, the four hallmark inflammatory response genes (*CD14*, *AQP9*, *SERPINE1*, and *ITGA5*) showed similar expression patterns as in GSE14520, i.e., downregulation of *CD14*, *AQP9*, and *SERPINE1* and upregulation of *ITGA5* (Figure 3(a)). Consistent with the GSE14520, patients in the high-risk group of the TCGA-LIHC dataset had significantly shorter OS than those in the low-risk group (hazard ratio = 1.910, 95%confidence interval = 1.343–2.716, *P* < 0.001, Figure 3(b)). Furthermore, IRPRS was found to be an independent prognostic factor compared to the routinely used clinicopathological characteristics (Figure 3(c)). In addition, we also explored the association between the IRPRS and the routinely used clinicopathological characteristics. The IRPRS showed no significant association with sex (Figure 4(a)), age (Figure 4(b)), serum alpha-fetoprotein (AFP) (Figure 4(c)), or Child-Pugh liver function level (Figure 4(f)). However, vascular invasion (Figure 4(d)), Eastern Cooperative Oncology Group (ECOG) performance status score (≥2) (Figure 4(e)), and advanced (III-IV) stage (Figure 4(g)) HCC were associated with high IRPRS. The IRPRS developed in this study could identify the high-risk subset of patients among those with serum AFP-negative HCC (Figure 4(h)). The IRPRS showed no association with GPC3 (Figure 4(i)), but was positively related with HSP70 (Figure 4(j)) and negatively related with GLUL (Figure 4(k)).

### 3.4. Potential Biological Characteristics of the High-Risk Group

The GSEA results indicated significant enrichment of many cancer-related hallmark gene sets in the high-risk group, such as epithelial-mesenchymal transition, hypoxia (Figure 5(a)), notch signaling (Figure 5(b)), angiogenesis (Figure 5(c)), and unfolded protein response (Figure 5(d)).

### 3.5. High- and Low-Risk Groups Showed Distinct Immune Microenvironment

The high-risk group showed greater numbers of various TILs (Figure 6), including regulatory T cells (Treg), B cells, CD4+ T cells, neutrophils, dendritic cells, macrophages, and NK cells. This reflects a more complex immune microenvironment of HCC in the high-risk group.

## 4. Discussion

The association between cancer and inflammation was first found in the nineteenth century, as cancers often occurred at sites of chronic inflammation and inflammatory cells were detected in cancer tissues [27]. It is estimated that approximately 20% of cancers may be induced by persistent infection or chronic inflammation [28]. A wide body of evidence has implicated inflammatory cytokines and inflammatory cells in the genesis and progression of HCC [1, 7, 8, 29]. In the present study, we proposed and validated an inflammatory response-related polygenic risk score for predicting prognosis of patients with HCC. The IRPRS was found to successfully categorize patients with HCC into two groups with distinct risk profile. Patients with high risk showed poorer prognosis than those with low risk. Furthermore, the IRPRS was an independent prognostic factor compared to the routine clinicopathological characteristics, including *α*-fetoprotein (AFP) levels and American Joint Committee on Cancer (AJCC) staging system. A high level of serum AFP is not only a diagnostic biomarker but also a confirmed biomarker of poor prognosis in all stages of HCC [30]. Although different thresholds of AFP have been reported [13, 31], it has been clearly demonstrated that patients with AFP > 400 ng/mL have poor outcomes [32]. However, approximately 30%–40% of patients with HCC show negative serum AFP [33, 34]. In addition, diagnostic and prognostic biomarkers based upon noninvasive criteria are currently challenged by the need for molecular information that requires tumor tissue. Our IRPRS for serum AFP-positive and AFP-negative HCC was not significantly different and could still identify the high-risk subset of patients with serum AFP-negative HCC. Thus, our IRPRS may be a promising prognostic tool for HCC, independent of AFP. Furthermore, the IRPRS was also independent of GPC3. Nevertheless, it is notable that the protein expressions of GPC3, HSP70, and GLUL detected using immunohistochemistry (and not the mRNA expressions) are considered diagnostic markers for HCC. Therefore, further study is required to assess the relation of IRPRS with these three markers.

Our IRPRS included four hallmark inflammatory response genes (*CD14*, *AQP9*, *SERPINE1*, and *ITGA5*). CD14 plays a dual role in tumorigenesis, which is associated with the activation of various signaling pathways in malignant cells or in TILs [35]. *AQP9* acts as a tumor suppressor in HCC through the Wnt/*β*-catenin pathway and inhibition of hypoxia-inducible factor 1*α* expression [36, 37]. *SERPINE1* contributes to the invasion, metastasis, and poor prognosis in HCC [38, 39]. It seems that *ITGA5* is an established oncogene in many cancers [40–42]. According to our present analysis, these four genes can form a reliable prognostic tool for HCC through effective weighting. Moreover, our GSEA results indicated to a certain extent the biological significance of the high-risk HCC identified by IRPRS. The high-risk HCC may be characterized by more severe hypoxia, more active angiogenesis, and EMT.

The immune microenvironment plays a pivotal role in the pathogenesis of HCC with approximately 90% of the HCC burden associated with prolonged hepatitis due to viral hepatitis, excessive alcohol intake, or NAFLD or NASH [43]. Previous studies in mice or humans suggest that HCC cells can generate an immune-tolerant, protumorigenic microenvironment [44, 45]. Our analysis indicated the cancer-promoting inflammatory responses may be more pronounced in the high-risk group. On the other hand, the high-risk group possessed a greater variety of TILs. Based on current evidence [46], the high-risk tumors with more infiltrating CD8 T cells may be more likely to benefit from immunotherapy. However, the increased Treg cells in the high-risk group may suppress the antitumor effect of CD8 T cells [47]. Higher infiltrating Treg was strongly associated with poor overall survival [48]. However, we may still have a long way to go before we fully understand the immune microenvironment in HCC. Notably, studies from mouse models report that virtually every type of immune cell may play both protumor and antitumor roles [24].

Although our present study may provide a novel prognostic tool for HCC, it has several notable limitations. Firstly, this IRPRS is proposed based on a retrospective study and needs to be validated or improved by prospective studies before its use in clinical practice. Secondly, the molecular mechanisms of these four genes in HCC are not yet fully understood; thus, it is not clear whether these genes are causal or merely prognostic markers in HCC. Thirdly, treatment exerts a significant influence on the prognosis of patients with HCC. Owing to the lack of treatment records in the datasets, our study failed to explore the relationship between treatment and IRPRS. Fourthly, we failed to identify the association between etiologies of liver disease and our IRPRS.

In conclusion, we identified and validated a four-hallmark inflammatory response gene-based polygenic risk score, which could successfully divide patients with HCC into high-risk and low-risk groups. These two risk groups of HCC possess significantly distinct prognostic and biological characteristics.

## Figures and Tables

**Figure 1:** The expression patterns of differentially expressed hallmark inflammatory response genes in hepatocellular carcinoma. (a) Volcano plot of differentially expressed hallmark inflammatory response genes. Red indicates upregulated genes and blue indicates downregulated genes. The four optimal hallmark inflammatory response genes are highlighted. (b) Hierarchical clustering dendrograms of the expression patterns of differently expressed hallmark inflammatory response genes that can distinguish HCCs and adjacent tissues.

**Figure 2:** The inflammatory response-related polygenic risk score in GSE14520. (a) Four hallmark inflammatory response genes were identified as optimal features in the least absolute shrinkage and selection operator Cox analysis. (b) Kaplan-Meier curve analysis indicating that patients in the high-risk group had significantly shorter overall survival than those in the low-risk group.

**Figure 3:** The inflammatory response-related polygenic risk score in TCGA-LIHC dataset. (a) The four hallmark inflammatory response genes show similar expression patterns as in GSE14520. (b) Kaplan-Meier curve analysis indicating that the patients in the high-risk group had significantly shorter overall survival than those in the low-risk group. (c) The IRPRS was an independent prognostic factor compared to the routine clinicopathological characteristics. AFP: *α*-fetoprotein; ECOG: Eastern Cooperative Oncology Group; AJCC: American Joint Committee on Cancer.

**Figure 4:** Correlation of the inflammatory response-related polygenic risk score (IRPRS) with the clinicopathological characteristics and three known biomarkers. The IRPRS in different (a) sex, (b) age, (c) serum *α*-fetoprotein (AFP) levels, (d) vascular invasion status, (e) Eastern Cooperative Oncology Group (ECOG) performance status, (f) Child-Pugh liver function levels, and (g) American Joint Committee on Cancer stages. (h) The prognostic value of IRPRS is observed in the subset of serum AFP-negative HCC. The IRPRS shows no association with (i) GPC3 and is positively related with (j) HSP70 and negatively related with (k) GLUL.

**Figure 5:** Various cancer-related hallmark gene sets enriched in the high-risk group, such as (a) epithelial-mesenchymal transition, hypoxia, (b) notch signaling, (c) angiogenesis, and (d) unfolded protein response.

**Figure 6:** Comparison of tumor-infiltrating lymphocytes (TILs) in high- and low-risk groups of hepatocellular carcinomas. aDC: autologous dendritic cells; pDC: plasmacytoid dendritic cells; iDC: interdigitating dendritic cells.

## Data Availability

The data for this study can be obtained from Gene Expression Omnibus (https://www.ncbi.nlm.nih.gov/geo/) and The Cancer Genome Atlas (https://portal.gdc.cancer.gov/).

## References

[1] Llovet J. M., Kelley R. K., Villanueva A. (2021). Hepatocellular carcinoma. *Nature Reviews Disease Primers*.

[2] Villanueva A. (2019). Hepatocellular carcinoma. *New England Journal of Medicine*.

[3] Giannini E. G., Farinati F., Ciccarese F. (2015). Prognosis of untreated hepatocellular carcinoma. *Hepatology*.

[4] Diakos C. I., Charles K. A., McMillan D. C., Clarke S. J. (2014). Cancer-related inflammation and treatment effectiveness. *The Lancet Oncology*.

[5] Lin L., Yan L., Liu Y., Qu C., Ni J., Li H. (2017). The burden of primary liver cancer and underlying etiologies from 2017 to 2015 at the global, regional, and national level: results from the global burden of disease study 2015. *JAMA Oncology*.

[6] Kanwal F., Kramer J., Asch S. M., Chayanupatkul M., Cao Y., El-Serag H. B. (2017). Risk of hepatocellular cancer in HCV patients treated with direct-acting antiviral agents. *Gastroenterology*.

[7] Alderton G. K. (2012). Inflammation: the gut takes a toll on liver cancer. *Nature Reviews Cancer*.

[8] He G., Karin M. (2011). NF-*κ*B and STAT3 - key players in liver inflammation and cancer. *Cell Research*.

[9] Racanelli V., Rehermann B. (2006). The liver as an immunological organ. *Hepatology*.

[10] Jakab L. (2015). The liver and the immune system. *Orvosi Hetilap*.

[11] Subramanian A., Tamayo P., Mootha V. K. (2005). Gene set enrichment analysis: a knowledge-based approach for interpreting genome-wide expression profiles. *Proceedings of the National Academy of Sciences*.

[12] Liberzon A., Birger C., Thorvaldsdottir H., Ghandi M., Mesirov J. P., Tamayo P. (2015). The Molecular Signatures Database (MSigDB) hallmark gene set collection. *Cell System*.

[13] Roessler S., Jia H.-L., Budhu A. (2010). A unique metastasis gene signature enables prediction of tumor relapse in early-stage hepatocellular carcinoma patients. *Cancer Research*.

[14] Ritchie M. E., Phipson B., Di Wu Y. H., Law C. W., Shi W., Smyth G. K. (2015). limma powers differential expression analyses for RNA-sequencing and microarray studies. *Nucleic Acids Research*.

[15] Tibshirani R. (1997). The lasso method for variable selection in the Cox model. *Statistics in Medicine*.

[16] Wu T. T., Chen Y. F., Hastie T., Sobel E., Lange K. (2009). Genome-wide association analysis by lasso penalized logistic regression. *Bioinformatics*.

[17] Friedman J. H., Hastie T., Tibshirani R. (2010). Regularization paths for generalized linear models via coordinate descent. *Journal of statistical software*.

[18] Mootha V. K., Lindgren C. M., Eriksson K. F. (2003). PGC-1*α*-responsive genes involved in oxidative phosphorylation are coordinately downregulated in human diabetes. *Nature Genetics*.

[19] Di Tommaso L., Destro A., Seok J. Y. (2009). The application of markers (HSP70 GPC3 and GS) in liver biopsies is useful for detection of hepatocellular carcinoma. *Journal of Hepatology*.

[20] Di Tommaso L., Franchi G., Park Y. N. (2007). Diagnostic value of HSP70, glypican 3, and glutamine synthetase in hepatocellular nodules in cirrhosis. *Hepatology*.

[21] Zhou F., Shang W., Yu X., Tian J. (2018). Glypican-3: a promising biomarker for hepatocellular carcinoma diagnosis and treatment. *Medicinal Research Reviews*.

[22] Wang C., Zhang Y., Guo K. (2016). Heat shock proteins in hepatocellular carcinoma: molecular mechanism and therapeutic potential. *International Journal of Cancer*.

[23] Tripathy K., Sodhi M., Kataria R. S., Chopra M., Mukesh M. (2021). In silico analysis of HSP70 gene family in bovine genome. *Biochemical Genetics*.

[24] Ringelhan M., Pfister D., O’Connor T., Pikarsky E., Heikenwalder M. (2018). The immunology of hepatocellular carcinoma. *Nature Immunology*.

[25] Aran D., Hu Z., Butte A. J. (2017). xCell: digitally portraying the tissue cellular heterogeneity landscape. *Genome Biology*.

[26] Charoentong P., Finotello F., Angelova M. (2017). Pan-cancer immunogenomic analyses reveal genotype-immunophenotype relationships and predictors of response to checkpoint blockade. *Cell Report*.

[27] Balkwill F., Mantovani A. (2001). Inflammation and cancer: back to Virchow?. *The Lancet*.

[28] Wang K., Karin M. (2015). Tumor-elicited inflammation and colorectal cancer. *Advances in Cancer Research*.

[29] Barash H., Gross E. R., Edrei Y. (2010). Accelerated carcinogenesis following liver regeneration is associated with chronic inflammation-induced double-strand DNA breaks. *Proceedings of the National Academy of Sciences*.

[30] Montal R., Andreu-Oller C., Bassaganyas L. (2019). Molecular portrait of high alpha-fetoprotein in hepatocellular carcinoma: implications for biomarker-driven clinical trials. *British Journal of Cancer*.

[31] Lv Y., Wei W., Huang Z. (2018). Long non-coding RNA expression profile can predict early recurrence in hepatocellular carcinoma after curative resection. *Hepatology Research*.

[32] Galle P. R., Forner A., Llovet J. M. (2018). EASL clinical practice guidelines: management of hepatocellular carcinoma. *Journal of Hepatology*.

[33] Taketa K. (1990). Alpha-fetoprotein: reevaluation in hepatology. *Hepatology*.

[34] Chen D.-S., Sung J.-L., Shed J.-C. (1984). Serum *α*-fetoprotein in the early stage of human hepatocellular carcinoma. *Gastroenterology*.

[35] Wu Z., Zhang Z., Lei Z., Lei P. (2019). CD14: biology and role in the pathogenesis of disease. *Cytokine & Growth Factor Reviews*.

[36] Qian Y., Liu F., Zhang W. (2020). AQP9 suppresses hepatocellular carcinoma cell invasion through inhibition of hypoxia-inducible factor 1*α* expression under hypoxia. *Journal of Gastroenterology and Hepatology*.

[37] Liao S., Chen H., Liu M. (2020). Aquaporin 9 inhibits growth and metastasis of hepatocellular carcinoma cells via Wnt/beta-catenin pathway. *Aging*.

[38] Zheng Q., Tang Z., Wu Z., Shi D., Song H. (1998). Inhibitor of plasminogen activator 1 (PAI-1) in hepatocellular carcinoma. *Zhonghua Wai Ke Za Zhi*.

[39] Jin Y., Liang Z. Y., Zhou W. X., Zhou L. (2020). Expression, clinicopathologic and prognostic significance of plasminogen activator inhibitor 1 in hepatocellular carcinoma. *Cancer Biomarkers*.

[40] Gong C., Yang Z., Wu F., Han L., Liu Y., Gong W. (2016). miR-17 inhibits ovarian cancer cell peritoneal metastasis by targeting ITGA5 and ITGB1. *Oncology Reports*.

[41] Zhang X., Cheng S.-L., Bian K. (2015). MicroRNA-26a promotes anoikis in human hepatocellular carcinoma cells by targeting alpha5 integrin. *Oncotarget*.

[42] Chen J., Ji T., Di Wu S. J., Zhao J., Lin H., Cai X. (2019). Human mesenchymal stem cells promote tumor growth via MAPK pathway and metastasis by epithelial mesenchymal transition and integrin alpha5 in hepatocellular carcinoma. *Cell Death & Disease*.

[43] Llovet J. M., Zucman-Rossi J., Pikarsky E. (2016). Hepatocellular carcinoma. *Nature Reviews Disease Primers*.

[44] Chiang D. Y., Villanueva A., Hoshida Y. (2008). Focal gains of VEGFA and molecular classification of hepatocellular carcinoma. *Cancer Research*.

[45] Horwitz E., Stein I., Andreozzi M. (2014). Human and mouse VEGFA-amplified hepatocellular carcinomas are highly sensitive to sorafenib treatment. *Cancer Discovery*.

[46] Juneja V. R., McGuire K. A., Manguso R. T. (2017). PD-L1 on tumor cells is sufficient for immune evasion in immunogenic tumors and inhibits CD8 T cell cytotoxicity. *Journal of Experimental Medicine*.

[47] Principe D. R., Chiec L., Mohindra N. A., Munshi H. G. (2021). Regulatory T-cells as an emerging barrier to immune checkpoint inhibition in lung cancer. *Frontiers in Oncology*.

[48] Wang X., Xiao Z., Gong J., Liu Z., Zhang M., Zhang Z. (2021). A prognostic nomogram for lung adenocarcinoma based on immune-infiltrating Treg-related genes: from bench to bedside. *Translational Lung Cancer Research*.

